The article "lncENST Suppress the Warburg Effect Regulating the Tumor Progress by the Nkx2-5/ErbB2 Axis in Hepatocellular Carcinoma" was retracted in 2023. Reasons: signs of a paper mill; compromised peer review; unreliable results or conclusions.

# lncENST Suppress the Warburg Effect Regulating the Tumor Progress by the Nkx2-5/ErbB2 Axis in Hepatocellular Carcinoma

**DOI:** 10.1155/2021/6959557

**Published:** 2021-12-06

**Authors:** Geng Chen, Jiayun Jiang, Xiaofei Wang, Kai Feng, Kuansheng Ma

**Affiliations:** ^1^Department of Hepatobiliary Surgery, Daping Hospital, Third Military Medical University (Army Medical University), Chongqing, China; ^2^Institute of Hepatobiliary Surgery, Southwest Hospital, Third Military Medical University (Army Medical University), Chongqing, China

## Abstract

The therapeutic efficacy of radiofrequency ablation (RFA) against liver cancer is often limited by proliferation and metastasis of residual tumor cells. These phenomena are closely associated with the Warburg effect, wherein ErbB2 is activated. While RFA inhibits the Warburg effect of residual tumor cells at the early stage, the specific mechanisms remain unclear. We explored the regulatory relationship between the long noncoding RNA ENST00000570843.1 (lncENST) and ErbB2 using lentiviral transfection of lncENST and ErbB2 overexpression/interference vectors in *in vitro* and *in vivo* models of hepatocellular carcinoma in the presence of sublethal heat at 50°C. ErbB2-mediated Warburg effect was suppressed by lncENST, as manifested by reduced glucose uptake and lactic acid production in SMMC-7721 cells. lncENST also increased tumor apoptosis and inhibited tumor progression in nude Balb/c mice for up to 28 days after RFA. Additionally, we predicted through bioinformatic analysis that the promoter of *ErbB2* binds to the transcription factor Nkx2-5, resulting in a negative regulatory effect. This speculation was confirmed by chromatin immunoprecipitation of the Nkx2-5 protein and *ErbB2*, indicating that ErbB2 transcription was curbed by Nkx2-5. We propose that lncENST downplays the Warburg effect in residual tumor cells by downregulating ErbB2 via Nkx2-5 activation. This study is aimed at providing molecular targets that can prevent residual tumor cell proliferation after RFA, with clinical significance in hepatocellular carcinoma treatment.

## 1. Introduction

Cancer-associated complications and deaths due to tumor progression, metastasis, and recurrence have become a critical clinical issue worldwide that lacks a comprehensive solution. Researchers and clinicians have been confronted with the challenge of developing fast, low-cost, and effective treatment schemes against various types of cancers, among which liver cancer or hepatocellular carcinoma (HCC) has one of the highest incident rates and mortality.

Radiofrequency ablation (RFA) is a minimally invasive technique that has been applied to treat HCC and has shown comparable results with surgical resection [1, 2]. Its main mechanism of action is to kill tumor cells by inducing a high temperature at the local tumor site. From the center to the peripheral region of the tumor, there is a gradual change in RFA temperature distribution, with the central area reaching a temperature of up to 300°C. However, at the transition zone of the tumor, RFA temperatures are in the range of 42–60°C [3]. While tumor cells in the central area are ablated effectively, those in the transition zone are not immediately eradicated. In this zone, though apoptotic mechanisms may be activated, a portion of residual tumor cells may recover their activity after sublethal heat shock, leading to post-RFA metastasis and recurrence of HCC [4, 5]. The incidence of residual cancer after insufficient RFA is reportedly 5–40%, which makes up a considerable portion of the population of cancer patients [6–8].

The article "lncENST Suppress the Warburg Effect Regulating the Tumor Progress by the Nkx2-5/ErbB2 Axis in Hepatocellular Carcinoma" was retracted in 2023. Reasons: signs of a paper mill; compromised peer review; unreliable results or conclusions.

The biological activities of residual cancer cells, such as proliferation, migration, and epithelial-mesenchymal transition, are often enhanced [9]. In particular, the Warburg effect pertains to cancer cells and has been a subject of highlight in recent cancer research trends. In brief, the process whereby cancer cells tend to metabolize through glycolysis rather than oxidative phosphorylation even in the presence of oxygen is known as the Warburg effect [10]. This metabolic reprogramming event promotes cancer cell growth and survival, but the molecular mechanisms implicated therein are complex and far from completely understood. Among the components involved in the Warburg effect, the oncogene *ErbB2*, also known as human epidermal growth factor receptor 2, was shown to exert the Warburg effect by activating heat shock factor 1 and in turn upregulating lactate dehydrogenase A [11]. Correspondingly, ErbB2 overexpression induced elevated glucose uptake and lactate production, indicating its prominent role in glucose metabolism and contribution to the metastatic potential of tumor cells [12].

We propose that altering the expression of oncogenes such as *ErbB2* may be a method of downplaying the metastatic potential of cancer cells caused by the Warburg effect. Combined with techniques such as RFA, this may offer a strategy to treat cancer effectively. The expression of oncogenes and tumor suppressors is related to the presence of a variety of factors, including the activation of various pathways [13, 14], DNA amplification [15], microRNAs and long noncoding RNAs (lncRNAs) [16, 17], and external stimuli [18]. Our preliminary studies revealed that when the expression of the lncRNA ENST00000570843.1 was silenced in HCC cells, the expression of the *ErbB2* gene was upregulated after RFA, suggesting that this specific lncRNA functioned to suppress the gene transcription of *ErbB2*. In addition, lncRNA ENST00000570843.1 (hereafter denoted as lncENST), among other lncRNAs, has interestingly been directly linked to sublethal heat treatment by RFA. In particular, RFA significantly increased the expression of lncENST in HCC cells [3], but the relationship between this phenomenon and ErbB2 activity is unknown.

The article "lncENST Suppress the Warburg Effect Regulating the Tumor Progress by the Nkx2-5/ErbB2 Axis in Hepatocellular Carcinoma" was retracted in 2023. Reasons: signs of a paper mill; compromised peer review; unreliable results or conclusions.

In summary, we speculate that lncENST has tumor suppressor properties and can be used in combination with RFA (50°C sublethal heat stress) to achieve the best effect of killing tumor cells by regulating the expression of ErbB2. We aimed to elucidate the detailed mechanism involved in RFA-mediated HCC suppression through lncENST overexpression, leading to downregulation of ErbB2 in vitro and in vivo. We further propose that lncENST directly binds and activates the transcription factor Nkx2-5, whose activity impairs the transcription of ErbB2 gene and downregulates ErbB2 protein expression, thereby inhibiting the Warburg effect in residual cancer cells.

## 2. Materials and Methods

### 2.1. Cell Culture and Lentiviral Transfection

The human HCC cell lines SMMC-7721 and LO2 were acquired from the China Center for Type Culture Collection and cultured in Dulbecco's modified Eagle medium (SH30022.01B, HyClone, South Logan, UT, USA) containing 10% fetal bovine serum (10270-106, Gibco, Grand Island, NY, USA). Cells were incubated in a humidified atmosphere with 5% CO_2_ at 37°C. The overexpression vector pCDH-CMV-MCS-EF1-CopGFP-T2A-Puro and interference vector pSICOR were purchased from Addgene (Watertown, MA, USA). lncENST and *ErbB2* were amplified through polymerase chain reaction (lncENST forward 5′-GCTCTAGAATAGCCGCCCGGCTAGCT-3′ and reverse 5′-CGGAATTCCCTTCCGGGTTCACGCTA-3′; *ErbB2* forward 5′-GCTCTAGAATGGAGCTGGCGGCCTTGTGC-3′ and reverse 5′-CGGAATTCTCACACTGGCACGTCCAGACC-3′) and inserted into the pLVX vector with EcoRI and BamHI restriction sites to produce lncENST and ErbB2 overexpression vectors (lnc-OV and ErbB2-OV, respectively). The interference fragment (lncENST 5′-GGAATTGTTGGTCAGGCAAAC-3′ and *ErbB2* 5′-GCTCTTTGAGGACAACTATGC-3′) was inserted into the pSICOR vector with XhoI and BamHI restriction sites to produce lncENST and ErbB2 interference vectors (lnc-INT and ErbB2-INT, respectively). SMMC-7721 cells were transfected with lnc-OV/INT or ErbB2-OV/INT using Lipofectamine 2000 (11668-027, Invitrogen, Carlsbad, CA, USA) according to the manufacturer's instruction. Nontransfected cells (labeled as “control”) were used as controls.

### 2.2. In Vitro Sublethal Heat Treatment and Nkx2-5 Activation

To simulate RFA, an *in vitro* sublethal heat stress model was established in SMMC-7721 cells. The cells were plated accordingly and stimulated in a heated water bath set to 50°C for 10 min. Thereafter, the treated cells were subjected to subsequent experiments immediately. To simulate the activation of Nkx2-5, a recombinant human Nkx2-5 protein (ab152305, Abcam, Cambridge, UK) was added at 2 *μ*g/mL.

The article "lncENST Suppress the Warburg Effect Regulating the Tumor Progress by the Nkx2-5/ErbB2 Axis in Hepatocellular Carcinoma" was retracted in 2023. Reasons: signs of a paper mill; compromised peer review; unreliable results or conclusions.

### 2.3. Cell Counting Kit-8 (CCK-8) Assay

A CCK-8 assay was conducted following the instructions provided with the assay kit (PAB180031, Bioswamp, Wuhan, China). Control or transfected SMMC-7721 cells were seeded into 96-well plates at 5 × 10^3^ cells/well in 100 *μ*L of growth medium and incubated overnight at 37°C. After the cells were subjected to sublethal heat treatment, 10 *μ*L of CCK-8 reaction mixture (included in the assay kit) was added to each well, and the cells were incubated for 4 h at 37°C. The absorbance of the wells was read using a microplate reader (Multiskan FC, Thermo Fisher Scientific, Waltham, MA, USA) at 450 nm.

### 2.4. Flow Cytometry for Apoptosis Detection

Cell apoptosis was assessed by flow cytometry using an FITC Annexin V Apoptosis Detection Kit I (556547, BD Biosciences, Franklin Lakes, NJ, USA) according to the manufacturer's instructions. Treated cells were trypsinized using 0.25% trypsin/ethylenediaminetetraacetic acid and centrifuged at 1000 × *g* for 5 min [19]. The supernatant was removed, and the cells were resuspended in phosphate-buffered saline (PBS) and counted. Approximately 1 × 10^6^ cells were then centrifuged at 1000 × *g* for 5 min at 4°C [19]. After the supernatant was discarded, 1 mL of precooled PBS was added to the cells to form a suspension, which was mixed and centrifuged at 1000 × *g* for 5 min at 4°C. The supernatant was removed and the previous step was repeated. Then, 200 *μ*L of binding buffer was added to the cells, and annexin V-fluorescein isothiocyanate and propidium iodide (5 *μ*L of each) were added to the cell suspension and gently mixed. The cells were incubated for 30 min at 4°C in the dark, and 300 *μ*L of binding buffer was then added; after which flow cytometry was performed immediately using a NovoCyte apparatus (ACEA Biosciences, Inc., San Diego, CA, USA) The data were analyzed using NovoExpress software (ACEA Biosciences, Inc.) [19].

### 2.5. Assessment of Glucose Uptake and Lactic Acid Production

Glucose uptake was evaluated using the Screen Quest™ Colorimetric Glucose Uptake Assay Kit (36503, AAT Bioquest, Sunnyvale, CA, USA) according to the manufacturer's instructions. Treated cells were incubated with 2-deoxyglucose at 37°C for approximately 30 min. The cells were then washed and lysed, and the cell lysate was incubated with the provided assay mixture at room temperature for 2 h. The absorbance was read at 570/610 nm and is indicative of the relative glucose uptake. For lactic acid production, a lactate assay kit (K607-100, BioVision, Milpitas, CA, USA) was applied following the manufacturer's instructions. The treated cells were seeded in 96-well plates at 50 *μ*L/well, and 50 *μ*L of reaction mixture containing 46 *μ*L of lactate assay buffer, 2 *μ*L of the probe, and 2 *μ*L of enzyme mix (all provided in the kit) was added to each well. The plates were mixed well and incubated at room temperature for 30 min in the absence of light. The absorbance was measured at 570 nm and is indicative of the relative lactic acid production.

The article "lncENST Suppress the Warburg Effect Regulating the Tumor Progress by the Nkx2-5/ErbB2 Axis in Hepatocellular Carcinoma" was retracted in 2023. Reasons: signs of a paper mill; compromised peer review; unreliable results or conclusions.

### 2.6. Quantitative Reverse Transcription Polymerase Chain Reaction (qRT-PCR)

RNA was extracted using TRIzol (15596026, Ambion, Inc., Foster City, CA, USA) and reverse-transcribed into cDNA using the RevertAid First Strand cDNA Synthesis Kit (K1622, Thermo Scientific) and TaqMan microRNA assay kit (Applied Biosystems, Foster City, CA, USA). qRT-PCR was performed using the SYBR Green PCR Kit (KM4101, KAPA Biosystems, Wilmington, MA) with the following primer sequences: ErbB2 forward 5′-ACCCGCTGAACAATACCA-3′ and reverse 5′-GGATCAAGACCCCTCCTT-3′; Nkx2-5 forward 5′-TGTGCGTCTGCCTTTCCC-3′ and reverse 5′-GCGTTGTCCGCCTCTGTC-3′; and GAPDH forward 5′-CCACTCCTCCACCTTTG-3′ and reverse 5′-CACCACCCTGTTGCTGT-3′. The experimental conditions were as follows: initial denaturation at 95°C for 3 min; 39 cycles of denaturation at 95°C for 5 s, annealing at 56°C for 10 s, and extension at 72°C for 25 s; and final extension at 65°C for 5 s and 95°C for 50 s. Data acquisition was carried out using the QuantStudio™ 6 Flex Real-Time PCR System (Applied Biosystems) and analyzed with the 2^-*ΔΔ*Ct^ method [19].

### 2.7. Western Blot

Total tissue or cellular proteins were isolated before WB assay. Cells were rinsed by cold PBS twice, followed by lysis using the radioimmunoprecipitation assay (RIPA) buffer (PAB180006, Bioswamp) under 4°C. Afterwards, cell samples were transferred to the Eppendorf tube, followed by 10 min of heating under 95°C and 10 min of centrifugation at 12000 × *g*. Thereafter, we obtained supernatants and preserved them under -80°C. Tissues (20 mg) were homogenized using RIPA buffer (150–250 *μ*L), followed by 15 min of centrifugation at 12000 × *g*. Afterwards, we harvested supernatants and preserved them under -80°C for subsequent analyses. The bicinchoninic acid assay kit (PAB180007, Bioswamp) was utilized to quantify protein contents in tissue and cellular supernatants in line with specific instructions. Then, protein sample aliquots (20 *μ*g) were separated by SDS-PAGE, followed by transfer onto PVDF membranes (IPVH00010, Millipore, Burlington, MA, USA) as well as blocking using PBS/Tween 20 (PBST) that contained 5% skimmed milk under ambient temperature for a 2 h period. Afterwards, we incubated membranes using primary antibodies under 4°C overnight, including rabbit anti-ErbB2 (PAB33179), anti-Nkx2-5 (PAB34145), or anti-GAPDH (PAB36264) antibodies (1 : 2000, Bioswamp for all). Membranes were later rinsed for 5 min using PBST thrice, followed by 1 h incubation using goat anti-rabbit IgG secondary antibody (1 : 20000, PAB160011, Bioswamp) under ambient temperature. After washing by PBST for 5 min thrice, immunodetection was carried out by the enhanced chemiluminescent reagent (WBKLS0010, Millipore). The Tanon-5200 system (Tanon, Shanghai, China) was employed for visualization, while Tanon software was used for analysis.

The article "lncENST Suppress the Warburg Effect Regulating the Tumor Progress by the Nkx2-5/ErbB2 Axis in Hepatocellular Carcinoma" was retracted in 2023. Reasons: signs of a paper mill; compromised peer review; unreliable results or conclusions.

### 2.8. Animal Experiments

All animal experiments were conducted in accordance with the ethical guidelines of the Hubei Province Animal Use and Protection committee (permit no. SYXK 2018-0104). Four-week-old female Balb/c-nu/nu mice (Huafukang Bioscience Co. Inc., Beijing, China) weighing 19–21 g was housed in a specific-pathogen-free environment. Before the experiment, the mice were anesthetized using 1% pentobarbital (30 mg/kg) via abdominal injection. The *in vivo* HCC xenograft model was established by injecting Huh-7 cells (1 × 10^7^ cells in 100 *μ*L for each mouse) subcutaneously into the right axillary region of the mice. After five days, the mice received tail vein injection of either lncENST or ErbB2 overexpression/interference lentiviral vectors (0.5 *μ*g/*μ*L in 20 *μ*L of saline for each mouse) once a week. Control mice were injected with saline only. For RFA treatment, a multipolar RFA apparatus (model TJ358 WE568, Shanghai Hongmai Medical Instrument Co., Ltd., Shanghai, China) was employed for the application of sublethal heat stress in the *in vivo* xenografted mice. RFA was performed once during the experimental period as previously described [20]. When the xenografted tumor has grown to a volume of 6 mm^3^, the needle probe of the RFA apparatus was inserted 5 mm into the tumor. RFA was applied at 2 W for 150 s at 300 J (RFA application under these conditions was able to reach a treatment radius of 4 mm). Tumor growth was monitored over 28 days by measuring the length and width of the tumor every other day. Tumor volume was calculated as volume = length × width^2^ ÷ 2. At the end of 28 days, the mice were sacrificed after anesthesia with 1% pentobarbital (30 mg/kg) via abdominal injection, and the tumors were extracted.

The article "lncENST Suppress the Warburg Effect Regulating the Tumor Progress by the Nkx2-5/ErbB2 Axis in Hepatocellular Carcinoma" was retracted in 2023. Reasons: signs of a paper mill; compromised peer review; unreliable results or conclusions.

### 2.9. Tissue Preparation and Embedding

Extracted tumor tissues were cut into small pieces (1.5 cm × 1.5 cm × 0.3 cm) and fixed in 10% formalin for 48 h. The fixed specimens were then washed with water and dehydrated in ethanol using a graded series of concentrations (50%, 70%, 85%, 95%, and 100%). Thereafter, the specimens were immersed in an equal volume of ethanol and xylene for 2 h and in pure xylene for another 2 h to be transparentized. Next, the specimens were embedded in melted paraffin wax for 3 h. The embedded tissues were cut with a rotary microtome (RM2235, Leica Biosystems, Buffalo Grove, IL, USA) into sections with a thickness of approximately 5 *μ*m.

### 2.10. Terminal Deoxynucleotidyl Transferase dUTP Nick End Labeling (TUNEL) Assay

Sectioned samples were immersed twice in xylene for 15 min each and washed with a graded concentration series of ethanol (100%, 95%, 85%, and 75%) for 5 min at each concentration. Then, the samples were washed with tap water for 10 min and incubated with proteinase K at room temperature for 15–30 min. A TUNEL reaction mixture was prepared using the components provided by the TUNEL assay kit (11684817910, Roche, Basel, Switzerland).

The tissue samples were incubated with 50 *μ*L of reaction mixture in a humidified environment at 37°C for 1 h and washed three times with PBS. Then, the samples were incubated with 50 *μ*L of peroxidase solution (provided in the kit) at 37°C for 30 min and washed three times with PBS. Thereafter, 50–100 *μ*L of diaminobenzidine was added to the samples and incubated at 15–25°C for 10 min. After three final washes with PBS, the samples were counterstained with hematoxylin (PAB180015, Bioswamp), dehydrated, transparentized, and sealed on coverslips. Apoptosis was visualized using an optical microscope, and apoptotic cells are stained in brown.

### 2.11. Immunofluorescence of Tissue Samples

Tissue sections were deparaffinized and subjected to antigen retrieval and endogenous peroxidase blocking as previously described. The sections were washed twice with PBST for 5 min each and blocked with 5% BSA for 10 min. After blocking, the sections were incubated with rabbit primary antibodies against ErbB2 (1 : 50, PAB33179, Bioswamp) or Nkx2-5 (1 : 50, PAB34145, Bioswamp) at 4°C overnight. The sections were washed three times with PBS for 5 min each and incubated with Alexa Fluor 488-conjugated Affinipure goat anti-rabbit IgG (H+L) secondary antibodies (1 : 200, PAB160027, Bioswamp) for 1 h at 37°C in the dark, followed by PBS washing for 3 × 5 min. Nuclear staining was carried out using 20 *μ*L of 4′,6-diamidino-2-phenylindole, and the samples were mounted on glass slides for fluorescence microscopy.

The article "lncENST Suppress the Warburg Effect Regulating the Tumor Progress by the Nkx2-5/ErbB2 Axis in Hepatocellular Carcinoma" was retracted in 2023. Reasons: signs of a paper mill; compromised peer review; unreliable results or conclusions.

## 3. Statistical Analysis

All experiments were performed in triplicates (*n* = 3), and the data are presented as the mean ± standard deviation (SD). Statistical analysis was carried out by one-way analysis of variance with Tukey's test for multiple comparisons using OriginPro 8. *p* < 0.05 is considered statistically significant.

## 4. Results

### 4.1. Sublethal Heat Accentuated the Effect of lncENST in Suppressing HCC Tumor Behavior

We first verified the role of lncENST in RFA-mediated HCC inhibition and the specific phenomena implicated therein. An *in vitro* model of HCC was established using SMMC-7721 cells, which were transfected with either lncENST overexpression (lnc-OV) or interference (lnc-INT) vectors (Figure 1(a)). Sublethal heat treatment was applied at 50°C to simulate RFA, and the growth behavior of transfected cells was monitored after heat stress. Heat-treated cells in which lncENST was silenced proliferated to a greater extent than did nontransfected cells, whereas those that overexpressed lncENST showed reduced proliferative ability (Figure 1(b)). The results of proliferation are complemented by apoptotic behavior (Figure 1(c)), whereby lnc-OV led to remarkable apoptosis (27.1%) in heat-treated cells and lnc-INT suppress the apoptosis (6.34%) compared to that of nontransfected cells (control, 9.4%).

We were interested in investigating whether these changes in proliferation and apoptosis were mediated by lncENST via the Warburg effect. Firstly, we evaluated the glucose uptake and lactic acid production, which are characteristic features of the Warburg effect, in sublethal heat-treated LO2 normal liver cells and HCC cells transfected with lnc-OV or lnc-INT. Evidently, the LO2 normal liver cells did not show a significant increase in glucose uptake (Figure 2(a)) and lactate production (Figure 2(b)). But the HCC cells wherein lncENST was silenced showed elevated levels of glucose uptake (Figure 2(c)) and lactic acid production (Figure 2(d)), whereas lncENST overexpression had an inhibitory effect on the two phenomena. In HCC-xenografted mice injected with lnc-OV, tumor growth slowed down substantially compared to that in nontreated mice, whereas lnc-INT promoted tumor growth to a large extent (Figure 2(e)). However, in all cases, RFA (black lines) showed therapeutic effect by reducing the tumor volume compared to that in non-RFA-treated mice (Figure 2(e)). We also compared the apoptosis of HCC cells in the xenografted tumors between various treatments by TUNEL assay. lnc-OV led to enhanced apoptosis (black arrows in Figure 2(f)), and after RFA, all tissues exhibited extensive areas of positive TUNEL staining (brown regions in Figure 2(f)), with lnc-OV showing the greatest degree of apoptosis. These observations suggested that the overexpression of lncENST exerted antitumor properties by suppressing the Warburg effect and tumor growth, and RFA accentuated these effects in conjunction with the administration of lnc-OV.

The article "lncENST Suppress the Warburg Effect Regulating the Tumor Progress by the Nkx2-5/ErbB2 Axis in Hepatocellular Carcinoma" was retracted in 2023. Reasons: signs of a paper mill; compromised peer review; unreliable results or conclusions.

### 4.2. ErbB2-Mediated Warburg Effect Was Attenuated in HCC Cells via Activation of Nkx2-5

Having established the link between lncENST and RFA-mediated HCC inhibition, we then verified the involvement of ErbB2 in promoting the Warburg effect. SMMC-7721 cells were transfected with either ErbB2 overexpression (ErbB2-OV) or interference (ErbB2-INT) vectors. Heat treatment was applied at 50°C to simulate RFA, after which glucose uptake (Figure 3(a)) and lactic acid production (Figure 3(b)) were assessed. We observed that when ErbB2 was overexpressed, both glucose uptake and lactic acid production were significantly increased. By contrast, both were decreased by ErbB2 interference. We then searched for factors that may induce or inhibit the expression of *ErbB2* at the transcriptional level. Bioinformatic analysis based on the Champion Chip Transcription Factor Search Portal from Qiagen [21] revealed that Nkx2-5 is a transcription factor that binds to the promoter region of the *ErbB2* gene. Thus, we added a recombinant Nkx2-5 protein to ErbB2-OV-transfected cells (to simulate Nkx2-5 activation) and monitored its effect on cellular metabolism. We observed that Nkx2-5 activation had an antagonistic effect on *ErbB2*, as its addition to ErbB2-OV-transfected cells induced lower glucose uptake and lactic acid production compared to those of cells that were only subjected to ErbB2-OV transfection. This may suggest the suppressive effect of Nkx2-5 on the Warburg effect by downplaying the function of *ErbB2* in cellular metabolism.

Next, we injected ErbB2-OV or ErbB2-INT into HCC-xenografted mice and examined whether they affected tumor growth behavior (Figure 3(c)). During the 28-day observation period, ErbB2-OV induced significant tumor growth, as indicated by the large increase in tumor volume compared with that in control mice. ErbB2-INT, on the other hand, did not seem to affect tumor growth. Application of RFA seemed to have an inhibitory effect on tumor growth, especially in ErbB2-OV-treated mice. In terms of tumor cell behavior, the TUNEL assay revealed many apoptotic cells when RFA was applied, especially after ErbB2-INT and ErbB2-OV treatment (Figure 3(d)). These observations implied that interference of ErbB2 alone did not influence tumor behavior drastically, but RFA was still able to effectively cause tumor cell death to a certain extent.

The article "lncENST Suppress the Warburg Effect Regulating the Tumor Progress by the Nkx2-5/ErbB2 Axis in Hepatocellular Carcinoma" was retracted in 2023. Reasons: signs of a paper mill; compromised peer review; unreliable results or conclusions.

### 4.3. lncENST Activated Nkx2-5 to Suppress Transcription of ErbB2

We proceeded to evaluate whether a targeting relationship exists between lncENST and ErbB2. After SMMC-7721 cells were transfected with lnc-OV or lnc-INT, they exhibited reduced and elevated mRNA expression of *ErbB2*, respectively (Figure 4(a)). Expectedly, ErbB2 protein expression followed the same trend (Figure 4(b)). *In vivo* experiments were also performed in nude mice subjected to tumor xenografts of HCC cells transfected with either lnc-OV or lnc-INT. The animals were accordingly treated with RFA, and ErbB2 expression was measured in tumor tissues. As anticipated, the RFA-treated tissues showed relatively lower mRNA and protein expression of ErbB2 than their nontreated counterparts, but in the same general tendency (Figures 4(c) and 4(d)).

Having established that lncENST has a negative regulatory effect on ErbB2, we investigated the mechanisms through which this occurs. We propose that sublethal heat-induced lncENST activates a certain intermediate factor that in turn controls the transcription of *ErbB2*. As previously indicated, the transcription factor Nkx2-5, which was predicted to bind to the promoter region of the *ErbB2* gene, diminished the effect of ErbB2 on cellular metabolism and downplayed the Warburg effect. To confirm our hypothesis, we assessed whether the expression of lncENST is related to that of Nkx2-5.  Figure 5(a) reveals that lnc-OV indeed upregulated the expression of Nkx2-5, whereas lnc-INT had the opposite effect, signifying the direct correlation between the expression of lncENST and Nkx2-5. We then aimed to complement the results that we have shown previously, which elucidated the relationship between lncENST and ErbB2, by integrating an activator of Nkx2-5 into the system to see whether it affected *ErbB2* expression. Though lnc-INT did not alter the mRNA expression of *ErbB2* significantly in Figure 5(b), the addition of an Nkx2-5 activator remarkably downregulated it compared to lnc-INT alone. Moreover, while the protein expression of ErbB2 was upregulated by lnc-INT, the activation of Nkx2-5 suppressed ErbB2 expression to levels similar to those induced by lnc-OV (Figure 5(c)), even when lncENST was silenced. Evidently, Nkx2-5 played antagonistic roles against lnc-INT by nullifying its upregulation of *ErbB2* and in turn greatly limiting ErbB2 protein expression. In other words, we can reasonably assume that lncENST and Nkx2-5 have complementary functions in mediating the transcription of *ErbB2*.

We subsequently observed the effect of Nkx2-5 on ErbB2 expression in tumor tissues from mice xenografted with lnc-OV/INT-transfected HCC cells by immunofluorescence (Figure 6(a)). After RFA treatment, the expression of ErbB2 was evidently increased in mice injected with lnc-INT but almost completely absent in those xenografted with lnc-OV. On the contrary, distinct expression of the transcription factor Nkx2-5 was observed in tumor tissues of lnc-OV-xenografted mice, while control and lnc-INT-xenografted mice showed minimal Nkx2-5 expression. Furthermore, lnc-OV decreased the mRNA expression of *ErbB2* in tumor tissues as it did in SMMC-7721 cells *in vitro*, while the mRNA expression of Nkx2-5 was decreased and increased by lnc-INT and lnc-OV, respectively (*p* < 0.05, Figure 6(b)). Evaluation of protein levels resulted in almost the same tendency in ErbB2 expression as that of mRNA expression, but whereas lnc-INT induced no change in *ErbB2* mRNA expression, it significantly increased the protein level of ErbB2 (*p* < 0.05, Figure 6(c)).

The article "lncENST Suppress the Warburg Effect Regulating the Tumor Progress by the Nkx2-5/ErbB2 Axis in Hepatocellular Carcinoma" was retracted in 2023. Reasons: signs of a paper mill; compromised peer review; unreliable results or conclusions.

Finally, we performed chromatin immunoprecipitation to confirm the prediction of bioinformatic analysis (Figure 6(d)), whereby a binding site between Nkx2-5 and the *ErbB2* gene was revealed. The interaction between the Nkx2-5 protein and the *ErbB2* gene was probed using an Nkx2-5 antibody to pull down the Nkx2-5/*ErbB2* complex after SMMC-7721 cells were transfected with overexpression or interference vectors of lncENST or Nkx2-5. The expression of *ErbB2* was then evaluated as an indication of transcriptional regulation (Figure 6(e)). Notably, we found that the overexpression of Nkx2-5 resulted in a reduction in *ErbB2* expression, suggesting that *ErbB2* transcription was hindered by Nkx2-5. However, in the absence of Nkx2-5, *ErbB2* expression was elevated immensely, further validating the regulatory effect of Nkx2-5 on the transcription of *ErbB2*.

## 5. Discussion

RFA is a safe yet powerful treatment for HCC that can act as an alternative or a complementary strategy to conventional surgical or chemotherapeutic methods. However, post-RFA residual tumor cells remain problematic as they may provoke recurrence and possess metastatic potential. The need to identify oncogenic or tumor-suppressing factors related to RFA treatment is thus apparent in order to increase its efficacy. We have previously reported that the expression of several lncRNAs was altered in HCC cells treated by sublethal heat [3], including the newly discovered lncRNA ENST00000570843.1 (lncENST). Considering the many discovered functions and activities of lncRNAs, it is unsurprising that they are vitally implicated in the regulation of tumor metabolism [22]. In residual HCC cells after insufficient RFA, the downregulation of the lncRNA FUNDC2P4 was demonstrated to enhance epithelial-to-mesenchymal transition by promoting E-cadherin expression. This phenomenon led to an increase in HCC proliferation, migration, and invasion, suggesting that the deficiency of FUNDC2P4 was associated with post-RFA HCC development and recurrence [23]. The functions and activities of lncENST, which was employed in our study, have not yet been reported in the literature. We sought to verify whether lncENST is a tumor suppressor that can be activated by RFA-induced sublethal heat and its activities in HCC cells. After subjecting lentivirus-transfected SMMC-7721 HCC cells to sublethal heat treatment at 50°C, we observed that lnc-OV restricted cell proliferation and promoted apoptosis (Figure 1). Because we aimed to elucidate the specific mechanism underlying these processes, we further examined factors that may be correlated with lncENST in affecting HCC cell metabolism to provide an explanation for the tumor-suppressing potential of lncENST.

The article "lncENST Suppress the Warburg Effect Regulating the Tumor Progress by the Nkx2-5/ErbB2 Axis in Hepatocellular Carcinoma" was retracted in 2023. Reasons: signs of a paper mill; compromised peer review; unreliable results or conclusions.

One of the important functions of lncRNAs is to facilitate cellular metabolism through a variety of enzymes and kinases. In this way, lncRNAs can influence glycolysis and have a direct impact on the Warburg effect in tumor cells [24]. This metabolic reprogramming subsequently promotes or suppresses malignant transformation, leading to tumorigenesis and cancer progression. For example, glycolysis was promoted in HCC cells by the lncRNA Ftx via the activation of peroxisome proliferator-activated receptor *γ*, resulting in tumor progression [25].

Conversely, the downregulation of the lncRNA IDH1-AS1 by the oncoprotein c-Myc contributed to the Warburg effect through hypoxia-inducible factor 1*α*, even in normoxic conditions [26]. We demonstrated herein that the overexpression of lncENST considerably reduced the expression of ErbB2, an oncogene that is known to trigger the Warburg effect [11]. The inhibition of glucose uptake and lactic acid production in HCC cells under sublethal heat stress in the presence of lnc-OV (Figures 2(a) and 2(b)) and ErbB2-INT (Figures 3(a) and 3(b)) validated this phenomenon. With this, we reasonably assumed that the antitumor effect of lncENST was related the restriction of the Warburg effect through suppressing ErbB2 expression. The *in vivo* experiments in HCC-xenografted mice also showed that sublethal heat treatment accentuated the tumor-suppressing effect of lncENST by promoting apoptosis and inhibiting the proliferation of tumor cells, as well as limiting tumor growth in lnc-OV-xenografted mice (Figures 2(c)–2(e)).

The targeting relationship between lncENST and ErbB2 was then clarified in our study in order to provide a mechanistic explanation of lncENST-mediated tumor suppression. Through bioinformatic analysis, we predicted that Nkx2-5 suppresses the transcription of the *ErbB2* gene by binding to its promoter region [21]. The homeobox transcription factor Nkx2-5 has critical functions in modulating cardiac growth [27] and has been implicated in heart defects and diseases [28, 29]. However, we suggest herein that Nkx2-5 may also participate in tumor-suppressing regulatory processes. We first showed that lnc-OV upregulated the expression of Nkx2-5, whereas lnc-INT downregulated it (Figures 5(a) and 5(b)). Notably, in both *in vitro* and *in vivo* experiments, lnc-INT did not seem to have a significant impact on the mRNA expression of *ErbB2*, whereas the corresponding protein expression of ErbB2 was substantially elevated by lnc-INT. This finding could be indicative of the prominent involvement of the transcription factor Nkx2-5 in regulating *ErbB2* activity. In particular, *ErbB2* is not necessarily affected by lncENST at the transcriptional level, but ErbB2 protein translation was directly influenced by the activation or inactivation of Nkx2-5 by lnc-OV or lnc-INT, respectively.

The article "lncENST Suppress the Warburg Effect Regulating the Tumor Progress by the Nkx2-5/ErbB2 Axis in Hepatocellular Carcinoma" was retracted in 2023. Reasons: signs of a paper mill; compromised peer review; unreliable results or conclusions.

The findings of our study can contribute to the development of optimized treatment schemes against various cancers, especially HCC. The shortcomings of RFA brought about by the presence of residual cancer cells can be addressed by combining gene therapy and other similar techniques. We highlighted the Warburg effect and suggested that altering or disrupting cellular metabolism could be a useful approach to incorporate. Herein, we demonstrated the important role of lncRNA ENST00000570843.1 in suppressing tumor growth by targeting and inhibiting ErbB2-mediated Warburg effect. As far as we know, lncRNA ENST00000570843.1 is a newly discovered lncRNA that has not been reported in any previous study other than ours. As such, the detailed properties and functions of lncRNA ENST00000570843.1 remain uncharacterized but could be of interest and warrant in-depth investigation. Given that the antitumor potential of this lncRNA has been revealed in the current study, we aim to further explore the properties of lncRNA ENST00000570843.1 in prospective studies, especially in terms of its interactions with oncogenes and therapeutic targets under various forms of stress and/or drug intervention. A comprehensive mechanistic understanding of the features and potential value of not only lncRNA ENST00000570843.1 but also other lncRNAs will allow us to take full advantage of their characteristics and harness their power in the next-generation development of anticancer strategies.

The newly discovered lncRNA ENST00000570843.1, which was upregulated by sublethal heat treatment, was demonstrated to negatively regulate the oncogenic protein ErbB2. The downregulation of ErbB2 in turn suppressed the Warburg effect in residual tumor cells to promote apoptosis and impair tumor progression in an HCC-xenografted mouse model. This process was associated with the activation of the transcription factor Nkx2-5, which was suggested to inhibit *ErbB2* expression via lncENST overexpression. In conclusion, the specific targets disclosed herein can be used as potential candidates for molecular and gene therapy for the development of treatment options for hepatocellular carcinoma.

The article "lncENST Suppress the Warburg Effect Regulating the Tumor Progress by the Nkx2-5/ErbB2 Axis in Hepatocellular Carcinoma" was retracted in 2023. Reasons: signs of a paper mill; compromised peer review; unreliable results or conclusions.

## Figures and Tables

**Figure 1:** Growth behavior of SMMC-7721 cells after transfection with lncENST interference or overexpression vectors. (a) lncENST transfection results. (b) CCK-8 detection of cell proliferation over a 72-hour period. The data are expressed as the mean ± SD, *n* = 3, ^∗^*p* < 0.05. (c) Flow cytometric analysis of cell apoptosis. The bottom and top percentage values represent the proportion of early and late apoptotic cells, respectively.

**Figure 2:** Effect of lncENST on cellular metabolism and tumor growth. The cellular metabolism of LO2 normal liver cells was evaluated by measuring (a) glucose uptake and (b) lactic acid production. The cellular metabolism of liver cancer cells was evaluated by measuring (c) glucose uptake and (d) lactic acid production, which are indicative of the Warburg effect. (e) Tumor growth in HCC-xenografted mice after lnc-INT/OV injection and RFA treatment. (f) Apoptosis of tumor tissues extracted from HCC-xenografted mice after lnc-INT/OV injection and RFA treatment. Positive staining is indicated in brown. Black arrows point to specific areas of positive staining. For (a)–(c), the data are expressed as the mean ± SD, *n* = 3, ^∗^*p* < 0.05. For (d), scale bar = 50 *μ*m, ×100.

**Figure 3:** Effect of ErbB2 on cellular metabolism and tumor growth. Cellular metabolism was evaluated by measuring (a) glucose uptake and (b) lactic acid production, which are indicative of the Warburg effect. (c) Tumor growth in HCC-xenografted mice after ErbB2-INT/OV injection and RFA treatment. (d) Apoptosis of tumor tissues extracted from HCC-xenografted mice after ErbB2-INT/OV injection and RFA treatment. Positive staining is indicated in brown. Black rectangles point to specific areas of positive staining. For (a)–(c), the data are expressed as the mean ± SD, *n* = 3, ^∗^*p* < 0.05. For (d), scale bar = 50 *μ*m, ×100.

**Figure 4:** Correlation between lncENST and ErbB2 *in vitro* and *in vivo*. Relative (a) mRNA and (b) protein expression of ErbB2 in SMMC-7721 cells subjected to lncENST interference or overexpression. Relative (c) mRNA and (d) protein expression of ErbB2 in tumor tissues of HCC-xenografted mice subjected to lnc-INT/OV injection and/or RFA treatment. For all, the data are expressed as the mean ± SD, *n* = 3, ^∗^*p* < 0.05.

The article "lncENST Suppress the Warburg Effect Regulating the Tumor Progress by the Nkx2-5/ErbB2 Axis in Hepatocellular Carcinoma" was retracted in 2023. Reasons: signs of a paper mill; compromised peer review; unreliable results or conclusions.

**Figure 5:** Involvement of Nkx2-5 in the targeting of ErbB2 by lncENST. (a) Relative protein expression of Nkx2-5 in SMMC-7721 cells subjected to lncENST interference or overexpression. Relative (b) mRNA and (c) protein expression of ErbB2 in SMMC-7721 cells transfected with lnc-INT/OV, with additional Nkx2-5 stimulus in lnc-INT-treated cells. For all, the data are expressed as the mean ± SD, *n* = 3, ^∗^*p* < 0.05.

**Figure 6:** Effect of Nkx2-5 on *ErbB2* expression in HCC-xenografted tumor tissues. (a) Immunofluorescence staining of ErbB2 and Nkx2-5 (punctate green dots in white rectangles) in tumor tissues of HCC-xenografted mice subjected to RFA and lnc-INT/OV injection. Scale bar = 50 *μ*m, ×100. Relative (b) mRNA and (c) protein expression of ErbB2 in tumor tissues of HCC-xenografted mice subjected to RFA and lnc-INT/OV injection. (d) Bioinformatic analysis based on the Champion Chip Transcription Factor Search Portal from Qiagen revealed the binding site between the transcription factor (TF in the image) Nkx2-5 and the *ErbB2* gene. (e) Chromatin immunoprecipitation of the Nkx2-5 protein and the *ErbB2* gene. Pull down was performed using an antibody against Nkx2-5. The expression of *ErbB2* was detected in SMMC-7721 cells treated with lnc/Nkx-OV/INT. For all, the data are expressed as the mean ± SD, *n* = 3, ^∗^*p* < 0.05.

## Data Availability

The data that support the findings of this study are available from the corresponding author upon reasonable request.
